# Construction of a Colorectal Cancer Prognostic Risk Model and Screening of Prognostic Risk Genes Using Machine-Learning Algorithms

**DOI:** 10.1155/2022/9408839

**Published:** 2022-10-11

**Authors:** Xuezhi Du, Han Qi, Wenbin Ji, Peiyuan Li, Run Hua, Wenliang Hu, Feng Qi

**Affiliations:** ^1^Department of General Surgery, Tianjin Medical University General Hospital, Tianjin Medical University, Tianjin 300052, China; ^2^College of Letters and Science, University of California, Berkeley, CA 94720, USA

## Abstract

This study is aimed at constructing a prognostic risk model for colorectal cancer (CRC) using machine-learning algorithms to provide accurate staging and screening of credible prognostic risk genes. We extracted CRC data from GSE126092 and GSE156355 of the Gene Expression Omnibus (GEO) database and datasets from TCGA to analyze the differentially expressed genes (DEGs) using bioinformatics analysis. Among the 330 shared DEGs related to CRC prognosis, we divided the analysis period into different phases and applied univariate COX regression, LASSO, and multivariate COX regression analysis. GO analysis and KEGG analysis revealed that the functions of these DEGs were primarily focused on cell cycle, DNA replication, cell mitosis, and other related functions, and this confirmed our results from a biological perspective. Finally, a prognostic risk model for CRC based on the CHGA, CLU, PLK1, AXIN2, NR3C2, IL17RB, GCG, and AJUBA genes was constructed, and the risk score enabled us to predict the prognosis for CRC. To obtain a comprehensive and accurate model, we used both internal and external evaluations, and the model was able to correctly differentiate patients with CRC into a high-risk group with poor prognosis and a low-risk group with good prognosis. The AUC values of the 3-, 5-, and 10-year survival ROC curves were 0.715, 0.721, and 0.777, respectively, according to the internal evaluation, and the AUC values were 0.606, 0.698, and 0.608, respectively, for the external evaluation using GSE39582 from the GEO database. We determined that CLU, PLK1, and IL17RB could be considered to be independent prognostic factors for CRC with significantly different expression (*P* < 0.05). Using machine-learning methods, a prognostic risk model comprised of eight genes was constructed. Not only does this model provide improved treatment guidance, but it also provides a novel perspective for analyzing survival conditions at a deeper biological level.

## 1. Introduction

Colorectal cancer (CRC) is one of the most widespread cancers worldwide and ranks third in regard to incidence and second in regard to mortality [1]. Moreover, the incidence and mortality rates for CRC have increased in recent years. Due to its atypical clinical symptoms, CRC can be detected in only 40% of the patients at an early stage [2]. Currently, the diagnosis of CRC is primarily based on colonoscopy, and its treatment involves surgery, radiotherapy, chemotherapy, targeted therapy, and immunotherapy. However, the prognosis for CRC differs among individuals. For example, the most common staging system for CRC is TNM staging. However, we observed that determining the prognosis of the patients at the same stage was very different [3]. The patients are often highly upset due to their poor prognosis.

It is important to predict the prognosis of patients with CRC. On one hand, it is possible that the patients may experience palindromia after surgery. If the prognosis of patients can be predicted, the group with a higher probability of palindromia development can be distinguished. Therefore, more attention should be focused on this group of patients to provide the necessary treatment. Dai et al. [4] constructed a prognosis risk model comprised of 15 mRNA and 3 lncRNAs. Their results indicated that the patients who are characterized as high risk exhibit a 2.7-fold greater risk for palindromia compared to that of the patients characterized as low risk. Therefore, it is important to construct an accurate model to predict the prognosis of patients with CRC.

However, after surgery, CRC may transfer to the liver or lung, and it is thus critical to identify the patients with poor prognosis and a higher probability of cancer metastasis. A recent study [5] identified 128 genes related to CRC EMT and constructed a risk model for metastasis. The results of this study indicated that for the patients in the Dukes' B stage, high-risk patients exhibit an 8.5-fold higher probability of metastasis compared to that of low-risk patients. In the Dukes' C stage, these patients exhibited a 3.6-fold higher probability. Therefore, it is highly recommended that high-risk patients should undergo chemotherapy, while low-risk patients do not need it, as chemotherapy is not beneficial to everyone due to its negative side effects. Consequently, constructing a risk model to group patients with CRC into high-risk and low-risk groups is important.

Scientists are searching for ways to detect poor prognosis early and to take action to prevent it [6–8]. Researchers have been attempting to understand the mechanisms of CRC. Unfortunately, this process is too complicated to be fully understood at the present time. Therefore, a new model is required to better predict CRC prognosis. We determined that prognosis may be related to the different gene expression profiles among individuals. Therefore, we aimed to determine the relationship between specific genes and CRC prognosis.

Certain studies have reported that right and left colon cancers may exhibit different prognoses [9]. Liang et al. [10] constructed a risk model based on PHACTR3 and CKMT2 to predict the prognosis of left-sided colon cancer. Additionally, there is another risk model based on EREG, ERFE, GFI1, and RASL10B specific for right colon cancer.

Gene sequencing techniques have greatly improved in recent years, and there are therefore numerous useful gene databases such as the Gene Expression Omnibus (GEO) and TCGA. With the help of the R language and machine learning, we can analyze a large amount of gene data and conclude their relationship with CRC. Algorithms such as COX regression and LASSO regression are commonly used in the context of bioinformatics research, and they can identify the most relevant and principal factors. We hope to combine them with certain gene data analysis techniques to determine the effects of genes on the prognosis of CRC.

In this study, we first identified differentially expressed genes (DEGS) in CRC using the GEO and TCGA databases. We obtained samples with survival data from the TCGA database. We then used univariate COX regression, LASSO regression, and multivariate COX regression to focus on special genes that exhibit a strong relationship with CRC and construct a prognostic risk model. Finally, we used the risk model to predict the prognosis of any sample from the above database. According to the survival curve and ROC curve of internal and external evaluations, our risk model was demonstrated to be effective.

## 2. Materials and Methods

### 2.1. Data Collection

All data used in this research were obtained from the GEO database (https://www.ncbi.nlm.nih.gov/geo/) and the Cancer Genome Atlas (TCGA) database (https://portal.gdc.cancer.gov/). We extracted CRC data from GSE126092 [11] and GSE156355 [12] of the GEO database and datasets from TCGA to analyze the differentially expressed genes. The GSE126092 dataset was uploaded in August 2020 and contained 10 CRC tissues and paired adjacent noncancerous tissues. GSE156355 was uploaded in February 2019 and contained six paired CRC samples and adjacent tissues. The datasets from the TCGA database contained 551 CRC tissues and 48 adjacent noncancerous tissues and provided survival information and living status. Finally, we used datasets from GSE39582 [13] in the GEO database to verify our risk model for external evaluation. GSE39582 was uploaded in May 2020 and contained data from 585 CRC tissues.

### 2.2. Selecting DEGs

All data were processed using R software (version 3.6.2). For GSE126092 and GSE156355, we first downloaded the series matrix files using GEOquery2.54.1. We then used the limma package (limma 3.42.2) to select DEGs with a threshold of |log2FC| > 1 and adjusted *P* < 0.05. We then downloaded the CRC data from the TCGA database. Based on a threshold of |log2FC| > 4 and adjusted *P* < 0.01, we selected the DEGs using the limma 3.42.2 package. Finally, we obtained three sets of DEGs from the three databases. Volcano plots were constructed using the ggplot2 3.3.2 package. We obtained the overlapping DEGs from these three datasets, and a Venn diagram was constructed using Venn Diagram 1.6.20.

### 2.3. Gene Sets Enrichment Analysis

#### 2.3.1. Gene Ontology (GO) Analysis

GO analysis [14] can provide information regarding the functions of genes. Our analysis revealed three aspects that included molecular function (MF), biological process (BP), and cellular component (CC). We used the R package clusterProfiler 3.14.3 to perform GO analysis of the DEGs based on these three aspects. Then, for each aspect, we selected the top 20 GO terms with the smallest *P* values. We used the R package GOplot 1.0.2 to plot the graph.

#### 2.3.2. Kyoto Encyclopedia of Genes and Genomes (KEGG) Pathway Enrichment Analysis

KEGG analysis [15] was also performed using the R package clusterProfiler 3.14.3 with a threshold of adjusted *P* < 0.05. The histogram was plotted using R package enrichplot 1.6.1.

### 2.4. Univariate COX Regression

The matrix files from the TCGA database contained 551 CRC tissues, and we finally obtained 509 useful examples after removing lost cases for follow-up. We used univariate COX regression to analyze the overlapping DEGs in step 2.2 to identify candidate genes that are relevant to survival. Candidate genes (*P* < 0.05) were retained for further analysis using the survival 3.1.8 package of the R language.

### 2.5. LASSO Regression

Next, we used LASSO regression to select genes related to CRC. LASSO regression is another regression model that can be used to analyze the relationship of various factors with a given phenomenon. From the results of the LASSO regression, factors with nonzero coefficients are more relevant. There is a predefined parameter (lambda) in the LASSO regression. As this parameter becomes larger, it is encouraged to use more zero coefficients for the factors. We first used cross-validation that represents a common means of selecting parameters in machine learning to select a suitable lambda value for our experiment. We then continued to screen relevant genes using the R packages glmnet 4.1 and survival 3.1.8.

### 2.6. Multivariate COX Regression

Finally, we used multivariate COX regression to analyze the 17 genes that were selected using LASSO regression in step 2.5. Let *X* = (*X*1, *X*2, ⋯, *X*17) be a vector of genes where *X1*, *X2*,…, *X17* are the differentially expressed genes identified in step 2.5. Let “*t*” be survival time. The variables used in our multivariate COX regression were *X* and *t*. Based on COX regression using R package survival 3.1.8, we obtained a coefficient for each gene and constructed the risk model using these coefficients. We can also plot a forest plot to illustrate the visual result of multivariate COX regression using the R package survminer 0.4.8.

### 2.7. Prognostic Risk Model for CRC

The risk model was applied to calculate the risk score based on the candidate genes and their coefficients that were obtained from multivariate COX regression. The formula is as follows:

(1) $$\begin{array}{c} \text{RiskScore}=\sum \left({{\text{coefGEN}}_{\text{i}}}^{*}\text{ expGE}{\text{N}}_{\text{i}}\right) \end{array}$$

where coefGEN_i_ is the coefficient value of each gene, and expGEN_i_ is the gene expression.

After calculating the risk scores for 509 samples in TCGA, we classified them into low-risk and high-risk groups according to the median risk score. The prognostic risk model was visualized using the R package pheatmap 1.0.12, and the risk score curve, survival time distribution map, and heatmap of prognostic genes for low-risk and high-risk groups were plotted.

### 2.8. Evaluation of the Risk Model

#### 2.8.1. Internal Evaluation

We used the median risk score as the cutoff and divided the 509 samples from TCGA into low- and high-risk groups. The survival curve was plotted using the K-M method with the R package survival 3.1.8. The ROC curve was plotted using a time ROC of 0.4, and the area under the ROC curves for 3 years, 5 years, and 10 years of survival were calculated.

#### 2.8.2. External Evaluation

Using the R package GEOquery 2.54.1, we downloaded datasets from GSE39582 of the GEO database and obtained 579 gene samples and survival data (six cases were lost). Similarly, we calculated the risk score for each sample using our risk model, used the median risk score as the cutoff, and divided these samples into low-risk and high-risk groups. Survival and ROC curves were plotted.

### 2.9. Identifying the CRC Prognostic Biomarkers

We used the genes in the above prognostic risk model as candidate genes and divided 509 samples in TCGA and 579 samples in GSE39582 into low- and high-risk groups, respectively, according to the median expression of each gene. The survival curves were plotted using the R package survival 3.1.8, and the candidate genes with *P* < 0.05 in both matrix files were identified as the final prognostic biomarker genes for CRC.

The total procedure in this study can be seen in Figure 1.

## 3. Results

### 3.1. Differentially Expressed Genes (DEGs) of CRC

We downloaded gene datasets for CRC tissues and paired adjacent noncancerous tissues from GSE126092, GSE156355, and TCGA. Volcano plots were used to visualize the DEGs in GSE126092 (Figure 2(a)), GSE156355 (Figure 2(b)), and TCGA (Figure 2(c)). Red dots represent upregulated genes, and blue dots represent downregulated genes. As presented in the results, there were 3,022 DEGs in GSE126092, 3,356 DEGs in GSE156355, and 3,926 DEGs in the TCGA dataset. Finally, 330 overlapping DEGs were identified in all three datasets as presented in the Venn diagram (Figure 2(d)). We will use these 330 DEGs in future studies.

### 3.2. Gene Sets Enrichment Analysis

GO and KEGG pathway analyses were performed to focus on the functions of these DEGs. We used R package GOplot 1.0.2 to plot graphs for GO analysis and enrichplot 1.6.1 for KEGG with the *y*-axis representing the term and the *x*-axis representing the number of genes. Color represents the *P* value. In the molecular function (MF) term, the top five functions that the DEGs were primarily enriched for were cyclin-dependent protein serine/threonine kinase regulator activity, catalytic activity acting on DNA, DNA helicase activity, 3′-5′ DNA helicase activity, and heparin binding (Figure 3(a)). In biological process (BP) term, the top five functions enriched by the DEGs were mitotic cell cycle checkpoint, sister chromatid segregation, cell cycle G1/S phase transition, negative regulation of mitotic cell cycle phase transition, and negative regulation of mitotic sister chromatid separation (Figure 3(b)). In the cellular component (CC) term, the top five functions that the DEGs were primarily enriched for were cyclin-dependent protein kinase holoenzyme complex, collagen-containing extracellular matrix, centromeric region of condensed chromosome, centromeric region of condensed nuclear chromosome, and chromosomal region (Figure 3(c)). KEGG pathway analysis indicated that these DEGs were primarily related to cell cycle pathways, DNA replication, mineral absorption, and progesterone-mediated oocyte maturation (Figure 3(d)).

### 3.3. Univariate COX Regression

Our goal was to analyze the relevance of different genes in the context of CRC. In our study, we identified 330 overlapping DEGs in step 2.2, and we analyzed 509 examples with survival times from the TCGA database. After univariate COX regression, we selected 42 genes with *P* < 0.05 as the inputs for the next step (Table 1). Among the 330 overlapping DEGs, there were 42 genes that were related to the prognosis of CRC.

### 3.4. LASSO Regression

We continued to analyze 42 genes related to prognosis and used LASSO regression to further select genes that exhibited a relatively stronger relationship with CRC. According to cross-validation, LASSO regression exhibited the highest prediction accuracy when lambda was the smallest (Figure 4(a)). We selected 17 genes with coefficients that were not zero in this model (Figure 4(b)). These genes were CALB2, SCG2, CHGA, FABP4, CLU, PLK1, MAD2L1, AGMAT, MIPEP, DSN1, AXIN2, PARM1, NR3C2, IL17RB, GCG, AJUBA, and ARHGAP44. These genes were more relevant in regard to CRC prognosis.

### 3.5. Multivariate COX Regression

We performed multivariate COX regression analysis using the 17 genes that were selected by LASSO regression. Finally, eight genes related to prognosis were selected according to the smallest Akaike information criterion (AIC) instead of the *P* value, and this ensured that we could obtain a more suitable risk model (Table 2).

Within these eight genes, if HR was greater than 1, then this gene was negatively related to the prognosis of CRC. Instead, if the HR was less than 1, it was positively related to prognosis. According to the results of the multivariate COX regression analysis, CHGA, CLU, GCG, and AJUBA were negatively correlated with prognosis, and PLK1, AXIN2, NR3C2, and IL17RB were positively correlated with prognosis (Figure 5(a)).

### 3.6. Visualization of the Prognostic Risk Model for CRC

Using multivariate COX regression, we obtained the prognostic risk model as follows (according to Equation (1)):

(2) $$\begin{array}{c} \text{RiskScore}=\left(0.00767*\exp CHGA\right)+\left(0.01449*\exp CLU\right)+\left(-0.05963*\exp\;PLK1\right)+\left(-0.01635*\exp AXIN2\right)+\left(-0.15748*\exp NR3C2\right)+\left(-0.03055*\exp IL17RB\right)+\left(0.02558*\exp\;GCG\right)+\left(0.07265*\exp\;AJUBA\right) \end{array}$$

where the coefficient for each gene was from Table 2 of the multivariate COX regression and was combined with gene expression.

Using this formula, we calculated the RiskScore for 509 samples from the TCGA database. The median RiskScore was used as the threshold value. Samples with higher values were in the high-risk group, and samples with lower values were in the low-risk group. We then plotted the risk score curve (Figure 5(b)) and survival time distribution map (Figure 5(c)) to visualize the prognostic risk model. There was a shorter survival time with an increasing risk score. The heatmap of prognostic genes for the low-risk and high-risk groups revealed differential expression of the eight target genes between the two groups (Figure 5(d)).

### 3.7. Evaluation of the Prognostic Risk Model for CRC

#### 3.7.1. Internal Evaluation

After calculating the RiskScore for 509 samples from the TCGA database and dividing the samples into low-risk and high-risk groups using the median score as the threshold value, there were 255 and 254 samples in the low-risk and high-risk groups, respectively. We then plotted survival curves (Figure 6(a)) for these samples. The average survival time for the high-risk group was much shorter than was that for the low-risk group, and this indicated that our risk model was effective (*P* = 3.018e − 06). We also plotted ROC curves for 3-, 5-, and 10-year survival (Figure 6(b)). The area under the curve (AUC) values were 0.715, 0.721, and 0.777, respectively.

#### 3.7.2. External Evaluation

We calculated the risk score for each sample from GSE39582. We also used the median score as the threshold value and divided the samples into low- and high-risk groups. There were 290 samples in the low-risk group and 289 samples in the high-risk group. We then plotted survival curves (Figure 6(c)) for these samples. The average survival time for the high-risk group was much shorter than was that for the low-risk group, and this indicated that our risk model was also effective for external data (*P* = 0.013). We then continued to plot the ROC curves for 3-, 5-, and 10-year survival (Figure 6(d)). The AUC values were 0.606, 0.698, and 0.608, respectively.

### 3.8. Identifying the CRC Prognostic Biomarkers

The samples in the TCGA database and in GSE39582 were divided into high-risk and low-risk groups with the median value of the expression of the eight genes involved in the above risk model used as cutoff values, and the survival curves for each gene were drawn separately. The expression of CLU, PLK1, and IL17RB were significantly different (*P* < 0.05) in both of the matrix files (Figures 7(a)–7(c)). CLU expression was negatively correlated with the survival of patients with CRC, while PLK1 and IL17RB expressions were positively correlated with survival time.

## 4. Discussion

CRC is a leading cause of death worldwide. Although much work has been performed, the incidence and mortality of CRC continue to increase. One of the primary reasons for this is the lack of precise diagnostic and prognostic biomarkers for CRC. One of the important pathogeneses of CRC is gene mutation and continuous accumulation, and these characteristics may serve as promising diagnostic and prognostic biomarkers [16]. In recent years, the beginning of the Human Genome Project and the development of high-throughput sequencing technology have enabled us to gain a deeper understanding of the pathogenesis of tumors, and at the same time, they have generated a large amount of sequencing data that has been followed by the emergence of databases such as TCGA and GEO databases to store these data. This has accelerated the application of bioinformatics in the context of tumors. Therefore, we can screen for biomarkers with diagnostic and prognostic functions by mining data in public databases, and we can then study their mechanisms of action.

R is a programming language that possesses a large number of extension packages that can achieve complex data processing, statistical analysis, graphic drawing, and other operations, and it possesses the advantage of being simple and easy to learn. Therefore, the R language can be used as a bridge between bioinformatics and medical research. In this study, the R language was used as a tool to screen for genes related to overall survival in CRC using machine-learning algorithms, and a prognostic risk model was constructed. The analysis process involves the processing of thousands of sample data points and the statistical analysis of tens of thousands of genes. Additionally, R packages allow us to display the analysis results with different legends such as volcano plots and Venn diagrams for differential genes, histograms for enrichment analysis, model risk score distribution plots, survival time and survival status plots, prognosis heatmaps of related genes, survival curve charts, and ROC curve charts for internal and external evaluation. The use of these legends visualizes complex data, makes them more concise and clearer, and fully reflects the advantages of bioinformatics methods in regard to the display of results.

We screened 330 genes that were differentially expressed between CRC tissues and adjacent tissues by joint analysis of CRC data from 509 samples from the TCGA database and from the GSE126092 and GSE156355 datasets. The functional enrichment analysis and KEGG pathway analysis demonstrated that the DEGs were primarily enriched in the functions of cell cycle, DNA replication, cell mitosis, and other related functions that were involved in the oncogenesis and progression of CRC. Univariate COX regression analysis revealed that among the 330 genes, there were 42 genes associated with overall survival in patients with CRC. LASSO regression analysis further screened for 17 genes that were associated with CRC prognosis. Multivariate COX regression analysis was performed on the genes in this group to determine the coefficients of each gene and to establish a prognostic risk model. Eight genes were selected for use in the prognostic risk model. Among these eight genes, the expression of CHGA, CLU, GCG, and AJUBA were negatively correlated with the overall survival of patients with CRC and were poor prognostic factors, and the expression of PLK1, AXIN2, NR3C2, and IL17RB were positively correlated with the prognosis of patients with CRC and were thus favorable prognostic factors.

The prognostic risk model for gene expression can predict the overall survival, recurrence, and metastasis risk of patients with cancer based on gene expression, and this is applicable in clinical settings. Certain gene-based risk models have emerged to differentiate the overall survival rate of the patients. Schetter et al. [17] established a prognostic risk model for cancer using inflammation-related genes. This study determined that the patients with high inflammatory risk scores exhibited increased cancer-related mortality, particularly in clinical stage II. In another study focused on a prognostic model consisting of LAMA1, ITGB1, ITGA2, CXCR4, and EGFA, the patients with high-risk scores tended to exhibit poor prognosis [18]. Zhou et al. determined a prognostic model consisting of five genes related to autophagy, divided the patients into high-risk and low-risk groups, and observed a significant difference in survival between the two groups. ROC analysis revealed that the 1-year and 3-year AUCs were 0.841 and 0.803, respectively, and the results were validated using an external validation set [19]. For our 8-gene prognostic risk model, we also performed internal and external evaluations of our eight-gene prognostic risk model. Internal evaluation in the TCGA database demonstrated that the prognostic risk model could significantly separate high-risk and low-risk patients. The ROC curves were drawn, and it was determined that the AUC values for 3-, 5-, and 10-year survival were all greater than 0.7, and this indicated a high prediction accuracy. In the external evaluation using GSE39582, the overall survival of high-risk patients was also significantly shorter than was that of low-risk patients with AUCs of 0.606, 0.698, and 0.608 for 3-, 5-, and 10-year survival, respectively. In the external evaluation, the AUCs of the three curves were slightly smaller than were those in the internal evaluation. Therefore, more data from different databases are required to confirm the validity of the risk model in the future.

Sequentially, we analyzed the expression of every gene involved in the above risk model with the median value as the cutoff value. CLU, PLK1, and IL17RB expression were significantly different as indicated by survival curves. The expression of CLU was negatively correlated with the survival of patients with CRC, while the expression of PLK1 and IL17RB was positively correlated with survival time.

Clusterin (CLU) is expressed in various tissues of the human body [20] and is a 449 amino acid, heterodimeric glycoprotein with a plausible role in the regeneration, migration, and antiapoptosis of tumor cells [21]. CLU can be detected in the serum of the patients with early stage CRC or hepatocellular carcinoma, and its expression gradually increases during CRC progression [22, 23]. The patients with high CLU expression exhibited worse prognosis [24]. Kim et al. [25] reported that silencing of CLU expression could downregulate survivin to thereby increase the sensitivity of nonsmall cell lung cancer to V-ATPase inhibitors, and it was proposed that PI3K/AKT/mTOR inhibitors combined with V-ATPase inhibitors may provide effective treatment for nonsmall cell lung cancer. A growing number of studies suggest that CLU can act as a target for colorectal cancer therapy, and high expression of CLU may indicate chemoresistance [26, 27].

Polo-like kinase 1 (PLK1) is a member of the well-conserved serine/threonine kinase family and is essential for tumor cell division and proliferation [28, 29]. PLK1 overexpression has been observed in many types of tumors, and therefore, PLK1 has long been considered as an oncogene [30]. However, the oncogenic properties of PLK1 have not been confirmed [31, 32]. In a study by de Cárcer et al. that was published in Nature Communications, PLK1 was speculated to act as a tumor suppressor rather than as an oncogene [33]. *In vivo*, Plk1 overexpression prevented the development of Kras-induced and Her2-induced mammary gland tumors in the presence of increased rates of chromosome instability. In the patients with specific breast cancer subtypes, PLK1 overexpression was correlated with improved survival. The effects of chromosome instability induced by PLK1 overexpression differ in different types of tumors. In colon cancer cells with partial APC gene knockout, PLK1 inhibits tumor growth [34]. TCGA data indicated that the patients with high PLK1 expression in lung adenocarcinoma, renal clear cell carcinoma, and bladder cancer exhibit shorter overall survival, whereas the patients with high PLK1 expression in squamous cell carcinoma, rectal cancer, and thymoma exhibit a better prognosis [35]. In our research, overexpression PLK1 in the context of CRC was associated with good prognosis.

Interleukin 17 receptor B (IL17RB) is a member of the IL17 receptor family and specifically binds to IL-17B and IL-17E (also known as IL-25) [36]. In breast cancer, high expression of IL17RB is associated with poor prognosis that is mainly the result of the interaction between IL-17B and IL17RB [37]. Moreover, recent work has demonstrated that elevated IL-17B is associated with poor prognosis in the patients with pancreatic, gastric, lung, and breast cancers [38, 39]. However, the combination of IL-17E and IL17RB exerted different effects. Studies have revealed that IL-17E inhibits the formation of breast cancer cell colonies expressing IL17RB *in vitro* [40]. Therefore, IL-17B can promote the growth of breast cancer tumor complexes in mice, while IL-17E can inhibit this process. Currently, there are few studies examining IL17RB in the context of CRC, and there are no relevant reports regarding the relationship between this receptor and overall survival of patients with CRC. Additionally, it remains unclear if IL17RB primarily acts through IL-17B or IL-17E in patients with CRC. Our study revealed that patients with CRC and high IL17RB expression exhibited a longer overall survival, and that IL17RB expression could be used as a good prognostic marker for CRC. This result requires further relevant studies to verify its accuracy in the future.

Our study possesses some limitations. The conclusions of this study are based on previous data from certain databases and require a prospective experiment designed to verify the conclusions or some of our own data to confirm them. The risk model established in this study only includes the overall survival of patients and other prognostic results such as recurrence and metastasis were not included in the analysis. They were also not analyzed in the context of other clinicopathological parameters. The specific behavior of these three genes as independent prognostic factors in CRC also must be confirmed by further studies.

## 5. Conclusions

In conclusion, this study screened the DEGs between CRC tissues and paired adjacent noncancerous tissues from the GEO and TCGA databases. Using the R language packages, we performed enrichment analysis for these DEGs to analyze their functions. Finally, we obtained a prognostic risk model for CRC containing eight target genes through machine-learning algorithms and performed internal and external validations for this model. We then revealed that the risk score could be used as a valuable independent prognostic indicator for patients with CRC, and that CLU, PLK1, and IL17RB could also be considered as independent prognostic factors for CRC.

## Figures and Tables

**Figure 1:** The overview of the procedure used in this study.

**Figure 2:** Identification of overlapping DEGs of CRC. (a) Volcano plot of DEGs in GSE126092 between CRC tissues and paired adjacent noncancerous tissues. A total of 3,022 DEGs were identified with red dots or blue dots in the plot. (b) Volcano plot of DEGs in GSE156355 identified 3,356 DEGs. (c) Volcano plot of DEGs in TCGA identified 3,926 DEGs. (d) Venn graph of overlapping DEGs among these three data sets. A total of 330 DEGs in all three independent cohorts were identified, and this indicated that these genes were present in all of the three datasets.

**Figure 3:** Gene sets enrichment analysis of overlapping DEGs in CRC. (a) Molecular function (MF) term for GO analysis. (b) Biological process (BP) term for GO analysis. (c) Cellular component (cc) term for GO analysis. (d) KEGG pathway analysis for DEGs.

**Figure 4:** LASSO regression for screening of prognosis related genes in CRC. (a) Cross-validation of LASSO regression for verifying the parameter lambda. (b) LASSO regression coefficient spectrum to screen for 17 genes that were more relevant to the prognosis of CRC.

**Figure 5:** Construction of the risk model for prognosis of CRC. (a) A visual result of multivariate COX regression analysis forest plot. CHGA, CLU, GCG, and AJUBA were negatively related to the prognosis when HR>1, and PLK1, AXIN2, NR3C2, and IL17RB were positively related to the prognosis when HR<1. (b) The risk score curve of 509 samples of TCGA, where the green curve indicates the low-risk group with lower RiskScore than the median risk score, and the red curve indicates the high-risk group with a higher RiskScore. (c) The survival time distribution map indicated that the patients with higher RiskScore values exhibited relatively shorter survival times and higher mortality rates (red dots indicate death). (d) The heatmap of prognostic genes for low-risk and high-risk groups where the 8 target genes were differentially expressed in different groups.

**Figure 6:** Evaluation of the prognostic risk model for CRC. (a) Survival curves of the high-risk group and the low-risk group for 509 samples from the TCGA (Internal data). The low RiskScore group (low-risk group) exhibited a longer survival time. (b) ROC curves for 3- (green curve), 5- (blue curve), and 10-year survival (red curve) for 509 CRC samples from the TCGA database. (c) Survival curves of high-risk group and low-risk group for GSE39582 (external data). The low RiskScore group (low-risk group) exhibited a longer survival time. (d) ROC curves for 3- (green curve), 5- (blue curve), and 10-year survival (red curve) for samples from GSE39582.

**Figure 7:** Survival curves of the high-risk group and the low-risk group for samples from the TCGA or GSE39582 that were divided by the median value of the expression of CLU, PLK1, IL17RB, respectively. (a) Survival curves of the high-risk group and the low-risk group for samples from the TCGA (left side, *P* = 0.029) or GSE39582 (right side, *P* = 0.027) that were divided by the median value of the expression of CLU. These values were negatively correlated. (b) Survival curves of the high-risk group and the low-risk group for samples from the TCGA (left side, *P* = 0.012) or GSE39582 (right side, *P* = 0.02) for PLK1. These values were positively correlated. (c) Survival curves of the high-risk group and the low-risk group for samples from the TCGA (left side, *P* = 0.002) or GSE39582 (right side, *P* = 0.004) for IL17RB. These values were positively correlated.

**Table 1:** Results of univariate COX regression.

Genes	HR	HR.95L	HR.95H	*P* value
CALB2	1.075168531	1.046511034	1.104610780	0.000000145
MMRN1	1.177992963	1.102176923	1.259024202	0.000001390
SCG2	1.136294207	1.075992885	1.199974964	0.000004380
CHGA	1.008260884	1.004368250	1.012168604	0.000030700
CADM3	1.471082666	1.193637511	1.813016254	0.000294669
FABP4	1.010864845	1.004320872	1.017451457	0.001109783
GPX3	1.013547500	1.005364841	1.021796757	0.001139274
CLU	1.013894313	1.005458670	1.022400730	0.001207801
RCAN2	1.162898316	1.060003479	1.275781183	0.001409139
PLK1	0.951773127	0.921575359	0.982960402	0.002658353
CCND1	1.010820410	1.003524380	1.018169485	0.003593027
MGP	1.005838658	1.001872497	1.009820521	0.003877044
SGCE	1.110563713	1.030969237	1.196303166	0.005713800
MFAP4	1.009969066	1.002762350	1.017227575	0.006628391
PRELP	1.034675030	1.008960246	1.061045192	0.007938749
MAD2L1	0.933275152	0.885218560	0.983940631	0.010461483
SFRP2	1.002566577	1.000574717	1.004562402	0.011530280
AGMAT	0.968625747	0.944791385	0.993061380	0.012151343
MIPEP	0.953418072	0.916549114	0.991770115	0.017756291
VSIG4	1.033985345	1.005547554	1.063227381	0.018835922
CCDC80	1.039974343	1.006339207	1.074733675	0.019455563
FHL1	1.029753094	1.004243700	1.055910468	0.021972453
DSN1	0.958530124	0.924293285	0.994035133	0.022468282
EPB41L3	1.135963669	1.016666636	1.269259178	0.024325247
AXIN2	0.989527226	0.980342126	0.998798384	0.026921215
HEXIM1	1.041947453	1.004470807	1.080822346	0.027903087
PARM1	0.988914084	0.978997996	0.998930610	0.030154696
CHRDL1	1.025388857	1.002373365	1.048932808	0.030416027
NR3C2	0.882165693	0.787326645	0.988428773	0.030731862
IL17RB	0.958795008	0.922419497	0.996604983	0.032982279
CDC45	0.942908559	0.893309918	0.995261032	0.032985263
GCG	1.017196705	1.001258421	1.033388700	0.034341311
AJUBA	1.095354855	1.006562312	1.191980113	0.034719811
WDR4	0.943248674	0.893260819	0.996033903	0.035465193
CCNB1	0.986749509	0.974543568	0.999108326	0.035690679
CRYAB	1.030028043	1.001890929	1.058955359	0.036291275
ARHGAP44	0.845014051	0.719943532	0.991812155	0.039344784
ADH1B	1.056282963	1.002144123	1.113346545	0.041375192
CCNA2	0.974828540	0.951169319	0.999076256	0.041983147
SRPK1	0.980350420	0.961688311	0.999374677	0.042995634
GNL3	0.983089244	0.966962682	0.999484758	0.043276128
OSBPL1A	1.108175856	1.001910012	1.225712602	0.045818190

HR: hazard ratio.

**Table 2:** Results of multivariate COX regression.

Genes	Coefficient	HR	*P* value
CHGA	0.00767	1.007729435	0.000758663
CLU	0.01449	1.014594124	0.019038662
PLK1	-0.05963	0.942115433	0.001248681
AXIN2	-0.01635	0.98378415	0.001317437
NR3C2	-0.15748	0.854291769	0.011767179
IL17RB	-0.03055	0.969911846	0.124412162
GCG	0.02558	1.025912125	0.002791552
AJUBA	0.07265	1.075349281	0.126224659

HR: hazard ratio.

## Data Availability

All data were obtained from the TCGA and GEO databases.
